# Fucoxanthin, a Marine Carotenoid, Suppresses *Mycoplasma pneumoniae*-Triggered Inflammatory Cytokine Production and Promotes Bacterial Clearance in a Murine Model

**DOI:** 10.1155/2022/6238162

**Published:** 2022-04-21

**Authors:** Hongbo Wu, Shu Li, Linlin Wang, Jun Liang, Lei Yan, Jianjiang Dong

**Affiliations:** ^1^Department of Pediatrics, Beijing Luhe Hospital, Capital Medical University, Beijing 100000, China; ^2^Department of Medical Function, Mudanjiang Medical University, Mudanjiang 157011, China; ^3^Department of Library, Mudanjiang Medical University, Mudanjiang 157011, China; ^4^Stem Cell Institute, Mudanjiang Medical University, Mudanjiang 157011, China; ^5^Department of Histology and Embryology, Mudanjiang Medical University, Mudanjiang 157011, China

## Abstract

*Mycoplasma pneumoniae* (MP), an atypical bacterium, is a common pathogenetic organism of respiratory infection in children. In the present study, we analyzed the beneficial role of fucoxanthin (Fx), a marine carotenoid, in a murine model of MP. C57BL/6 mice were inoculated once intranasally with 10^7^ CFU of *M. pneumoniae*, and we found that Fx treatment markedly decreased BAL (quantitative bronchoalveolar lavage) *M. pneumoniae* concentrations and alleviated airway obstruction in the infected mice. Moreover, the concentrations of proinflammatory cytokines, including IL-6, TNF-*α* and IL-1*β*, were significantly decreased by Fx treatment in the BAL samples of infected mice. In vitro study further indicated that Fx treatment markedly suppressed the production of proinflammatory cytokines in mouse peritoneal macrophages after *M. pneumoniae* infection. In conclusion, this may be the first study to report the protective role of Fx against *M. pneumoniae* infection, providing a potential therapeutic agent for MP.

## 1. Introduction

Mycoplasmas are the smallest (50–300 nm in diameter) free-living organisms. *Mycoplasma pneumoniae* (MP) is recognized as a worldwide cause of community-acquired pneumonia in children and young adolescents [1]. MP in children is an acute lung inflammation caused by atypical *Mycoplasma* infection, accounting for about 10%–40% of community-acquired pneumonia in children. In clinical manifestations, severe complications such as bronchiectasis, necrotizing pneumonia, even fatal pneumonia, and damage of multisystem function may occur in children with MP infection. In this situation, the therapeutic effect is poor and the hospitalization time is prolonged [2]. The strong inflammatory responses induced by *M. pneumoniae* are closely related to the pathogenic factors to induce pneumonia [3]. Thus, there is an urgent need to identify more appropriate methods to alleviate inflammatory responses in MP.

In recent years, natural products draw great attention from scientists around the world. Fucoxanthin (Fx; Figure 1(a)), a natural product of carotenoids, is widely recognized as a potential drug source obtained from marine algae [4]. This compound has a wide range of pharmacological properties, including antioxidant, anti-inflammatory, and antimicrobial activities [5, 6]. Fx also attenuates LPS-induced acute lung injury and ameliorates the inflammatory responses [7]. The objective of the present study was to determine the beneficial role of Fx in a murine model of MP, as well as the related underlying mechanisms.

## 2. Materials and Methods

### 2.1. *M. pneumoniae* Preparation

*M. pneumoniae* wild-type (WT) strain M129, obtained from American Type Cell Collection (Manassas, VA, USA), was cultured in SP4 broth in culture flasks at 37°C. After 72 h, *M. pneumoniae* were harvested by centrifugation and resuspended in PBS solution to achieve a concentration in the range of 10^8^–10^9^ CFU/ml. Aliquots were stored at −80°C.

### 2.2. Animals and Treatments

Forty male C57BL/6 mice, purchased from Shanghai Laboratory Animal Center (Shanghai, China), were housed under a 12-hour light/dark cycle in a temperature-controlled room (22–24°C). The animals were supplied with water and standard chow ad libitum. All animal care and experimental protocols were approved by the ethics committee of hospital. All efforts were made to minimize animal suffering.

Fx (purity ≥95% by HPLC) was purchased from Sigma-Aldrich (St. Louis, MO, USA) and dissolved in DMSO before use.

The mice were allowed to acclimate to new environment for 1 week and then randomized into four groups (*n* = 10/group). On day 0, the mice in group A were treated with 100 *μ*l vehicle solution (PBS solution containing 25 mM HCl) by nasal drops, while the mice in group C and group D were successively given Fx orally at a dose of 50 mg/kg for five days. Then, the mice in group B and group D were inoculated intranasally infected with *M. pneumoniae* M129 (10^7^ CFU in 50 *μ*l of SP4 broth) on day 1. On day 5, the mouse lungs were lavaged with 1 ml of sterile saline. Cell-free bronchoalveolar lavage (BAL) fluid samples were stored at –80°C. Whole-lung specimens (including the trachea and both lungs) were collected, fixed in buffered formalin, dehydrated in 70% ethanol, cut in 4 *μ*m thick sections, and stained with hematoxylin and eosin. Morphometric analysis was performed under an optical microscope.

### 2.3. Measurement of Cytokine Production

The concentrations of IL-6, TNF-*α*, and IL-1*β* in culture supernatants were measured using specific ELISA kits (Affymetrix-eBioscience, Santa Clara, CA, USA), according to the manufacturer's instructions.

### 2.4. Cell Culture and Treatments

Peritoneal macrophages were isolated from male C57BL/6 mice, as previously described [8]. The isolated macrophages were seeded into 6-well plates and cultured in the RPMI-1640 medium (HyClone, Logan, UT, USA), containing 10% fetal bovine serum (FBS; HyClone) at 37°C in a humidified incubator with 5% CO_2_.

Cells in group A were treated with vehicle (DMSO). Cells in group C and group D were treated with 20 *μ*M Fx. After 2 h, cells in group D were infected with *M. pneumoniae* (20 CFU/ml) for another 24 h. Cells in group B were infected with *M. pneumoniae* (20 CFU/ml) for 24 h without Fx treatment.

### 2.5. Statistical Analysis

All statistical analyses were carried out using GraphPad Prism 6.0 software (GraphPad Software, Inc., La Jolla, CA, USA). The data were expressed as the mean ± standard deviation (SD). Differences among two or more independent groups were analyzed using Student's *t*-test or one-way analysis of variance followed by Tukey's test. *P* values of less than 0.05 were considered as statistically significance.

## 3. Results

All abbreviations and their full names are given in Table 1.

As shown in Figure 1(b), the concentration of MP was observed in the BAL samples of mice in groups A and C. After comparison, it was found that the concentration of MP in the BAL samples of mice in group B was significantly higher than that in group A (*P* < 0.05); the concentration of MP in the BAL samples of mice in group D was significantly lower than that in group B (*P* < 0.05).

As shown in Figure 2, the lung histomorphology of mice in groups A and C was normal, the lung tissues of mice in group B showed significant pathological changes of alveolar wall thickening and bronchial stenosis, while the inflammatory infiltration status in the lung tissues of mice in group D was significantly alleviated.

Figure 3 shows that the concentrations of IL-6, TNF-*α*, and IL-1*β* in BAL samples of group B were significantly higher than those of group A (*P* < 0.05); the concentrations of IL-6, TNF-*α*, and IL-1*β* in BAL samples of group D mice were significantly lower than those of group B (*P* < 0.05); there was no statistically significant difference in the concentrations of IL-6, TNF-*α*, and IL-1*β* in BAL samples of groups A and C (*P* > 0.05).

Figure 4 shows that the concentrations of IL-6, TNF-*α*, and IL-1*β* in peritoneal macrophages of group B were significantly higher than those of group A (*P* < 0.05); the concentrations of IL-6, TNF-*α*, and IL-1*β* in peritoneal macrophages of group D were significantly lower than those of group B (*P* < 0.05); there was no statistically significant difference in the concentrations of IL-6, TNF-*α*, and IL-1*β* in peritoneal macrophages of groups A and C (*P* > 0.05).

## 4. Discussion

MP is a community-acquired infection occurring mainly in children. Drug development for MP is still a tough challenge. Previous studies have shown that inoculation with *M. pneumoniae* induces significant airway obstruction in mice [9]. Consistent with this, in the present research, we successfully established the murine model of MP, and we observed that Fx treatment could promote the clearing of *M. pneumoniae* infection and protect the mouse lung from *M. pneumoniae*-induced injury, as evidenced by the alleviation of airway obstruction.

The pathogenesis of MP infection is attributed to an excessive immune response, and cytokine content is closely related to the severity of MP [10]. Zhao et al. [11] concluded that IL-6 level in bronchoalveolar lavage fluid in children with severe MP was significantly higher than that in children with mild MP, indicating that IL-6 is closely related to the severity of MP. The changes in the contents of proinflammatory cytokines IL-6, TNF-*α*, and IL-1*β* in BAL samples from MP-infected mice were examined using ELISA, and it was found that the levels of proinflammatory factors in BAL samples from MP mice were significantly higher than those from normal mice, while Fx treatment significantly decreased the concentrations of proinflammatory cytokines. Macrophages are one of the major immune cells that internalize MP during infection [12]. Collins et al. [13] demonstrated that TNF-*α* levels significantly increased in MP-infected mice and their macrophages. Vitro analysis also confirmed that Fx treatment significantly inhibited the production of proinflammatory cytokines IL-6, TNF-*α*, and IL-1*β* in peritoneal macrophages of mice after MP infection. In conclusion, to our knowledge, this may be the first study to report the protective role of Fx against *M. pneumoniae* infection, providing a potential therapeutic reagent for MP.

## 5. Conclusions

In order to investigate the inflammatory response and the therapeutic effect of Fx after MP infection, the MP mice model was obtained by MP pathogen infection, and Fx was used for the treatment of mice. The results showed that the lung tissues of MP mice had obvious pathological changes, and the contents of proinflammatory cytokines IL-6, TNF-*α*, and IL-1*β* in bronchoalveolar lavage fluid and macrophages were significantly increased. However, after treatment with Fx, the histopathological changes and proinflammatory factor levels in the lungs of MP mice were significantly improved. The above results confirmed that Fx can play a protective role after MP infection by reducing the inflammatory response of the body. The results can provide a reference for the research and development and selection of new drugs for the clinical treatment of MP.

## Figures and Tables

**Figure 1:** (a) The chemical structure of fucoxanthin (Fx). (b) The concentrations of *M. pneumoniae* in the BAL samples of mice. ^*∗*^*P* < 0.05 vs. group A; ^#^*P* < 0.05 vs. group B.

**Figure 2:** The pathological changes in lung tissues of mice.

**Figure 3:** The concentrations of proinflammatory cytokines in the BAL samples of mice. ^*∗*^*P* < 0.05 vs. group A; ^#^*P* < 0.05 vs. group B.

**Figure 4:** The concentrations of proinflammatory cytokines in the mouse peritoneal macrophages. ^*∗*^*P* < 0.05 vs. group A; ^#^*P* < 0.05 vs. group B.

**Table 1:** Abbreviations and full names.

Abbreviation	Full name
MP	*Mycoplasma pneumoniae*
Fx	Fucoxanthin
CFU	Colony forming unit
BAL	Bronchoalveolar lavage
IL-6	Interleukin-6
TNF-*α*	Tumor necrosis factor-*α*
IL-1*β*	Interleukin-1*β*
WT	Wild-type
PBS	Phosphate buffer solution
DMSO	Dimethyl sulfoxide
ELISA	Enzyme-linked immunosorbent assay
FBS	Fetal bovine serum
RPMI	Roswell Park Memorial Institute
SD	Standard deviation

## Data Availability

The data used to support the findings of this study are available from the corresponding author upon request.

## References

[1] Atkinson T. P., Balish M. F., Waites K. B. (2008). Epidemiology, clinical manifestations, pathogenesis and laboratory detection of mycoplasma pneumoniae infections. *FEMS Microbiology Reviews*.

[2] Wood P. R., Kampschmidt J. C., Dube P. H. (2017). Mycoplasma pneumoniae and health outcomes in children with asthma. *Annals of Allergy, Asthma & Immunology*.

[3] Shimizu T. (2016). Inflammation-inducing factors of mycoplasma pneumoniae. *Frontiers in Microbiology*.

[4] D’Orazio N., Gemello E., Gammone M., de Girolamo M., Ficoneri C., Riccioni G. (2012). Fucoxantin: a treasure from the sea. *Marine Drugs*.

[5] Liu M., Li W., Chen Y., Wan X., Wang J. (2020). Fucoxanthin: a promising compound for human inflammation-related diseases. *Life Sciences*.

[6] Karpiński T. M., Adamczak A. (2019). Fucoxanthin-an antibacterial carotenoid. *Antioxidants*.

[7] Li X., Huang R., Liu K. (2020). Fucoxanthin attenuates LPS-induced acute lung injury via inhibition of the TLR4/MyD88 signaling axis. *Aging*.

[8] Zhang X., Goncalves R., Mosser D. M. (2008). The isolation and characterization of murine macrophages. *Current Protocols in Immunology*.

[9] Fonseca-Aten M., Ríos A. M., Mejías A. (2005). Mycoplasma pneumoniaeInduces host-dependent pulmonary inflammation and airway obstruction in mice. *American Journal of Respiratory Cell and Molecular Biology*.

[10] Xu X.-F., Li X.-J., Liu J.-L., Wu L., Chen Z.-M. (2016). Serum cytokine profile contributes to discriminating M. pneumoniae pneumonia in children. *Cytokine*.

[11] Zhao J., Li Y., Zhang W. (2020). The clinical significance of IL-6s and IL-27s in Bronchoalveolar lavage fluids from children with mycoplasma pneumoniae pneumonia. *BMC Infectious Diseases*.

[12] Athamna A., Kramer M. R., Kahane I. (1996). Adherence ofMycoplasma pneumoniaeto human alveolar macrophages. *FEMS Immunology and Medical Microbiology*.

[13] Collins K. L., Younis U. S., Tanyaratsrisakul S. (2021). Angiotensin-(1-7) peptide hormone reduces inflammation and pathogen burden during mycoplasma pneumoniae infection in mice. *Pharmaceutics*.

